The article "End-to-End Autonomous Exploration with Deep Reinforcement Learning and Intrinsic Motivation" was published in 2021. Journal: Comput Intell Neurosci.

# End-to-End Autonomous Exploration with Deep Reinforcement Learning and Intrinsic Motivation

**DOI:** 10.1155/2021/9945044

**Published:** 2021-12-16

**Authors:** Xiaogang Ruan, Peng Li, Xiaoqing Zhu, Hejie Yu, Naigong Yu

**Affiliations:** ^1^Faculty of Information Technology, Beijing University of Technology, Beijing, China; ^2^Beijing Key Laboratory of Computational Intelligence and Intelligent System, Beijing, China

## Abstract

Developing artificial intelligence (AI) agents is challenging for efficient exploration in visually rich and complex environments. In this study, we formulate the exploration question as a reinforcement learning problem and rely on intrinsic motivation to guide exploration behavior. Such intrinsic motivation is driven by curiosity and is calculated based on episode memory. To distribute the intrinsic motivation, we use a count-based method and temporal distance to generate it synchronously. We tested our approach in 3D maze-like environments and validated its performance in exploration tasks through extensive experiments. The experimental results show that our agent can learn exploration ability from raw sensory input and accomplish autonomous exploration across different mazes. In addition, the learned policy is not biased by stochastic objects. We also analyze the effects of different training methods and driving forces on exploration policy.

## 1. Introduction

Exploration behavior is the fundamental of organisms for survival and reproduction. For example, animals searching for food may have to travel long distances without getting any reward from the environment [1, 2]. Likewise, autonomous exploration is essential for many applications in robotics [3, 4] and has garnered increased interest in recent years.

Autonomous exploration is challenging because the agent must localize itself, recognize explored areas, and plan a route to cover the environment. This work considers agents that need to explore the environment through vision. For traditional exploration methods, agents require a tabular representation of the environment and rely on the Q-value of state-action pairs to complete the exploration. The Q-value size is determined by the number of times the agent visits the pair and the Q-learning algorithms. Although some later studies have nicely balanced the exploration-exploitation problem [5, 6], the classical methods cannot be applied in high-dimensional state spaces because they had no way to cope with dimensional catastrophes. Recent deep reinforcement learning (DRL) [7], which combines deep convolutional neural networks (CNNs) and reinforcement learning (RL) [8], provides a framework for learning control policy for specific tasks. DRL has achieved impressive results in many robotic tasks [9–11], including methods that attempt to finish autonomous exploration from raw sensory input.

There have been many research efforts to make exploration techniques more suitable for high-dimensional state spaces. Bellemare [12] proposed a pseudocount method that generalizes a count-based method to the nontabular case. This approach improves the agent's exploration efficiency in a number of hard games, particularly Montezuma's Revenge. Ostrovski et al. [13] used a Pixel CNN model to supply pseudocount and achieved outstanding performance in many Atari games. In addition, this research discovered that the mixed Monte Carlo update is a powerful facilitator for exploration. Tang et al. [14] integrated the hash table with the classic count-based method to compute the novelty bonus of state. This combination allowed the method to reach near state-of-the-art performance on various continuous DRL benchmarks. Houthooft et al. [15] introduced an exploration method that rewards the agent by maximizing information about the agent's belief in environment dynamics. This method achieves superior performance in simple video games but struggled in complex environments. Relying on the theory that novel states are easier to distinguish than others, Fu et al. [16] used an exemplar model to detect novelty during interaction and combine it with a count-based method to guide exploration in egocentric observations. Pathak et al. [17] proposed an intrinsic curiosity module (ICM) that compute reward based on the prediction error. The ICM pushed the agent in ViZDoom and Super Mario Bros to explore the environment more efficiently, but it did not work when the agent observed something unpredictable. Burda et al. [18] took prediction error as a reward signal and conducted a large-scale study of purely curiosity-driven learning. The experiment results show a high alignment of behavior guided by curiosity-driven intrinsic motivation and hand-designed extrinsic reward in many game environments. Furthermore, this work discusses the limitations of prediction-based curiosity methods that have no way to deal with curiosity traps caused by unpredictable objects. Savinov et al. [19] created curiosity through a reachability network and episode memory [20]. This method solves navigation problems in sparse reward environments and overcomes the “couch-potato” issues in prior works, which manifests as agents being attracted to unpredictable objects and stopping exploration, but it cannot guide the agent to finish autonomous exploration in no-reward environments. Some navigation methods use auxiliary tasks, such as reward prediction [21], depth prediction, and loop closure classification [7], to encourage the agent to explore the environment faster.

In this study, we propose a DRL method, augmented with intrinsic motivation, for training agents to accomplish autonomous exploration through vision only. Considering the limitations in prediction-based exploration methods, we calculate the intrinsic motivation based on the episode memory. To accomplish the objective of covering the environment, we use two methods of generating intrinsic motivation. The first is a count-based method, which pays attention to the novelty bonus of the environment that has been explored and encourages the agent to reach the rarely visited states. The second method is determined by temporal distance [22, 23] between current observation and those in memory. It calculates the novelty bonus of unexplored areas and tries to push the agent to distant places. In our approach, the intrinsic motivation is a combination of such novelty bonuses. This enables our approach to outperform existing methods and achieves substantial scalability. We further analyze the role of different training methods and driving forces on learning exploration policy.

The rest of the paper is structured as follows: in Section 2, the background to our approach is listed. In Section 3, the architecture and algorithm details are introduced. In Section 4, the proposed algorithm is simulated and experimentally tested, and the test results are analyzed and discussed. Finally, the conclusions and future work are given in Section 5.

## 2. Background

### 2.1. Reinforcement Learning Foundation

Standard RL assumes the agent interacts with the environment in a number of discrete time steps. At each time step *t*, the agent observes a state *s*_*t*_(*s* ∈ *S*) and selects an action *a*_*t*_(*a* ∈ *A*) according to its policy *π*, where *π* is a mapping from states to actions. In return, the agent enters the next state *s*_*t*+1_ and receives a scalar reward *r*_*t*_. The process continues until the maximum time steps of an episode or reaches a terminal state. The reward *R*_*t*_=∑_*k*=0_^*∞*^*γ*^*k*^*r*_*t*+*k*_ is the accumulated return from the time step *t* with the discount factor *γ* ∈ (0,1]. The goal of the agent is to maximize expected return from each state *s*_*t*_, and there are two common ways to do this: value-based and policy-based methods.

The value function *V*^*π*^(*π*)=Ε[*R*_*t*_*|s*_*t*_=*s*] is the expected return for following policy *π* from state *s*, and the more familiar action-value function *Q*^*π*^(*s*, *a*)=Ε[*R*_*t*_*|s*_*t*_=*s*, *a*] is defined as the expected return for selecting action *a* in state *s* and following policy *π*. In many RL approaches, the action-value function is represented with a function approximator, and the famous one is DQN [24], which aims to approximate the optimal action-value function through CNNs. In contrast to value-based method, policy-based method directly parameterize the policy *π*(*a|s*; *θ*) and update the parameter *θ* by gradient ascent on Ε[*R*_*t*_]. One example of such an algorithm is REINFORCE [25], which updates the policy parameter *θ* in the direction ∇_*θ*_log  *π*(*a*_*t*_*|s*_*t*_; *θ*) [26].

As described above, the ultimate goal of the value-based method is the same as the policy-based method, but they use different way to obtain the policy, and each of them has its respective pros and cons. In order to combine the merit of both, the Actor-Critic (AC) [27] algorithm is proposed. Inside the framework, the actor and critic are represented by policy *π* and value function *V*^*π*^(*s*_*t*_), respectively, and the advantage estimation *A*(*s*_*t*_, *a*_*t*_)=*Q*(*s*_*t*_, *a*) − *V*(*s*_*t*_) is used to scale the policy gradient. The running diagram of the AC algorithm is shown in Figure 1, it is an iterative optimization process, and the two blue lines represent the time difference (TD) errors used to update the “Actor” and “Critic,” respectively.

### 2.2. Asynchronous Advantage Actor-Critic Algorithm

The asynchronous advantage actor-critic (A3C) [28] algorithm is an online DRL method. It maintains a policy *π*(*a*_*t*_*|s*_*t*_; *θ*) and a value function *V*(*s*_*t*_; *θ*_*v*_) during interaction and relies on parallel actor-learners to provide accumulated update. Like the variant of n-step Q-learning, A3C also operates in the forward view and uses the same mixed n-step return to update policy and value function after every *t*_max_ actions until a terminal state being reached. The update is performed by the estimation of an advantage function *A*(*s*_*t*_, *a*_*t*_; *θ*, *θ*_*v*_) given by *R*_*t*_ − *V*(*s*_*t*_; *θ*_*v*_), where *R*_*t*_=∑_*i*=0_^*k*−1^*γ*^*i*^*r*_*t*+*i*_+*γ*^*k*^*V*(*s*_*t*+*k*_; *θ*_*v*_) and *k* ∈ (0, *t*_max_]. In addition, although the parameter *θ* of policy *π*(*a*_*t*_*|s*_*t*_; *θ*) and *θ*_*v*_ of value function *V*(*s*_*t*_; *θ*_*v*_) are computed and updated separately, sharing some parameters and adding entropy regularization terms have been shown to be helpful for learning control policy.

In the A3C algorithm, each agent independently interacts with the environment. Due to the randomly initialized parameters, the observed states, the selected actions, and the achieved reward are different between agents, which is shown in Figure 2, thus enabling asynchronous update and reducing the relevance of training samples. Similar to other nonsynchronous methods, the loss function of the policy and value function is calculated by the following equations, respectively:

(1) $$\begin{array}{c} f_{\pi }\left(\theta \right)=\log\;\pi \left(a_{t}|s_{t};\theta \right)\left(R_{t}-V\left(s_{t};\theta_{v}\right)\right), \end{array}$$

(2) $$\begin{array}{c} f_{v}\left(\theta \right)={\left(R_{t}-V\left(s_{t};\theta_{v}\right)\right)}^{2}. \end{array}$$

The losses of every learner are collected in terms of the standard noncentered RMSProp, as shown in (3) and (4), to update the global network. After each update, the global network transmits the policy and value function to each actor.

(3) $$\begin{array}{c} g=\alpha g+\left(1-\alpha \right)\nabla \theta^{2}, \end{array}$$

(4) $$\begin{array}{c} \theta \;\leftarrow \;\theta -\frac{\eta \nabla \theta }{\sqrt{g+\varepsilon }}, \end{array}$$

where *g* is the moving average of elementwise squared gradients, 0 ≤ *α* ≤ 1 is a hyperparameter, *η* is the learning rate, and *ε* is the constant added to maintain numerical stability.

### 2.3. Nav A3C Model

The Nav A3C model [7] is an end-to-end navigation framework that incorporates multiple objective. Similar to A3C, Nav A3C maximizes accumulated return through actor-critic architecture and uses policy *π*(*a*_*t*_*|s*_*t*_; *θ*) and value function *V*(*s*_*t*_; *θ*_*v*_) to select actions.

The architecture details of Nav A3C are shown in Figure 3. Nav A3C has a three-layer-CNN encoder and uses a stacked LSTM to address the memory requirement. The inputs to this model include the agent observation *o*_*t*_ ∈ *R*^3×*W*×*H*^ (where *W* and *H* are the width and height of the image, respectively), the velocity *v*_*t*_ ∈ *R*^6^, the previous action *a*_*t*−1_ ∈ *R*^*N*_*A*_^, and the previous reward *r*_*t*−1_ ∈ *R*. Inside the model, the first LSTM layer receives the reward, and the velocity and previously selected action are directly fed to the second recurrent layer. The policy and value function share all intermediate representation, and each of them is computed by linear layer.

## 3. Exploration Method

In this section, we introduce the temporal correlation network, explain how to create intrinsic motivation based on episode memory, and then describe the exploration model.

### 3.1. Temporal Correlation Network

The temporal correlation network (TC-network, *ϕ*_*TC*_) is trained to compute the temporal distance between observations, a process critical for creating intrinsic motivation.

Conceptually, we use TC-network to accomplish a classification task. The network is trained to assign high similarity to pairs of observation that are temporally close and low similarity to pairs that are temporally distant. The TC-network architecture, shown in Figure 4, consists of two parts: an embedding part *ϕ*_*E*_ that is constructed based on ResNet-18 [29] and calculates the raw observations (*o*_*i*_, *o*_*j*_) into feature vectors and a comparator part*ϕ*_*C*_ that takes features as input and output the temporal correlation coefficient *tc* between observations:

(5) $$\begin{array}{c} tc=\phi_{TC}\left(o_{i},o_{j}\right)=\phi_{C}\left(\phi_{E}\left(o_{i}\right),\phi_{E}\left(o_{j}\right)\right). \end{array}$$

The training samples of TC-network are in a triple form 〈*o*_*i*_, *o*_*i*+*k*_, *y*_*ik*_〉, consisting of two observations and a binary label. These observations are considered close (*y*_*ik*_=1) if they are separated by at most *k* steps. Negative examples are pairs where the two observations are separated by at least *M* • *k* steps where the hyperparameter *M* is necessary to create a gap between positive and negative examples. In the end, the network is trained with logistic regression loss to output the probability of the positive class.

### 3.2. Formulate Intrinsic Motivation

It is difficult for one agent to act near-optimally until it has sufficiently explored the environment. The key question, however, is how to generate such exploration behavior. Obviously, relying on simple entropy maximization as a source of actions is difficult in complex environments, and annotating each environment with a hand-designed dense reward is not scalable. Inspired by the cognitive mechanism in animals, the intrinsic motivation method [30] is proposed. Such methods use a curiosity-driven intrinsic reward to guide exploration behavior. Theorists in many fields suggested the patterns of intrinsic motivation include empowerment [31], surprise [32], and novelty [33]. The way we make up intrinsic motivations is based on the novelty theory, which shows that an animal has the ability to reward itself for something novel. Our intrinsic motivation includes two types of novelty bonuses, both related to the episode memory.

The first part of our intrinsic motivation is calculated based on count-based method. For models that use the same approach, the novelty of a state-action pair is derived from the number of times an agent has reached that pair. Such approaches require an enumerable representation of the environment to prevent the dimension explosion problems which prevents the count-based method being practical for high-dimensional state spaces. Our approach discretizes the state space by TC-network *ϕ*_*TC*_ : *S*⟶*M* and uses the stored observations (*o*^*m*^ ∈ *M*) to represent the environment. States are mapped to a memory buffer. So, their occurrences can be counted by corresponding observations within memory. Then, these counts are used to calculate reward according to the classic count-based method, and such novelty bonus *r*^*cb*^ : *S*⟶*R* is defined as

(6) $$\begin{array}{c} r^{cb}\left(o^{c},o^{m}\right)=\frac{\alpha }{\sqrt{n\left(\phi_{TC}\left(o^{c},o^{m}\right)\right)}}, \end{array}$$

where *α* ∈ *R*_≥0_ is the bonus coefficient, *o*^*c*^ is the current observation, and *o*^*m*^ is the observations stored in memory. For every mapping *o*^*c*^⟶*o*^*m*^(*o*^*m*^ ∈ *M*) being found, the corresponding *n*(*ϕ*_*TC*_(*o*^*c*^, *o*^*m*^)) is increased by one. Certainly, the count-based method can effectively calculate the novelty bonus of current state when the mapping is discovered. However, if the mapping is not existing, in other words, if the current observation is in the unexplored part of environment, it is difficult to calculate the reward.

As previously mentioned, an animal can reward itself when it sees something novel, but the size of the reward varies with the effort that the agent has made. This intuition can be formalized as giving a reward to observations that are outside the already explored part of the environment, and the size of the reward is proportional to the shortest temporal distance between the current observation and those in memory. Therefore, the other part of our intrinsic motivation *r*^*t*  *d*^ : *S*⟶*R* is defined as

(7) $$\begin{array}{c} r^{t\;d}\left(o^{c},o^{m}\right)=\underset{o^{m}\in M}{\min}\left\{\frac{\beta }{\phi_{TC}\left(o^{c},o^{m}\right)}\right\}, \end{array}$$

where *β* ∈ *R*_≥0_ is the bonus coefficient, *o*^*c*^ is the current observation, and *o*^*m*^(*o*^*m*^ ∈ *M*) is the observations stored in memory. The intrinsic motivation *r*^*i*^(*o*^*c*^, *o*^*m*^) is defined as the sum of the two types of novelty bonuses:

(8) $$\begin{array}{c} r^{i}\left(o^{c},o^{m}\right)=r^{cb}\left(o^{c},o^{m}\right)+r^{t\;d}\left(o^{c},o^{m}\right). \end{array}$$

The process for calculating intrinsic motivation is depicted in Figure 5. To determine the novelty bonus of the current observation, we must keep track of the explored region, and the memory buffer is a good choice for that. However, we cannot store every observation during the interaction because such actions may make the current observation always temporally close to the previous step. In our method, the current observation is added to memory only if *r*^*i*^ is larger than the novelty threshold *r*^th^. This operation induces a discretization in the memory, thus ensuring the temporally distant observations are stored. As a side benefit, the memory buffer stores information with low redundancy.

### 3.3. Exploration Model

The exploration model is shown in Figure 6. Its main body is constructed based on the Nav A3C model and adjusted according to the exploration task. The most obvious change occurs in the architecture of the encoder and memory unit. First of all, to reduce the complexity of training, our method uses a two-layer CNN encoder and outputs 16 and 32 features, respectively, instead of a three-layer CNN encoder and 32 and 64 features in the Nav A3C model. Since our method does not need to store additional environment information provided by auxiliary tasks, the 1 layer LSTM is able to meet the memory requirement. The input to this model includes the observation *o*_*t*_ ∈ *R*^3×*W*×*H*^ (where *W* and *H* are the width and height of the image), the previous action *a*_*t*−1_ ∈ *R*^|*A*|^, and the previous reward *r*_*t*−1_^*i*^ ∈ *R*. At every time step *t*, the action *a*_*t*_ is selected to maximize the reward *r*_*t*_^*i*^. It should be noted that, in addition to the two types of novelty bonus generated by the agent itself, the reward *r*_*t*_^*i*^ does not include any reward from the environment. We use the A3C algorithm with n-step lookahead value to update policy *π*(*a*_*t*_*|s*_*t*_; *θ*) and value function *V*(*s*_*t*_; *θ*) and use an entropy regularization penalty to discourage premature convergence. During training, many instances of agent interact in parallel with many instances of environment.

## 4. Experiment

In this section, we evaluate the performance of our method in exploration task and compare it to relevant baselines.

### 4.1. Experiment Setup

#### 4.1.1. Experiment Environment

We test our approach and relevant baselines in multiple mazes from DMLab [34]; the illustration of an agent navigating toward a goal in the environment is shown in Figure 7. In this 3D simulation environment, the agent perceives the environment from a first-person perspective and have access to additional environmental information such as inertial information and local depth information. The action space is discrete while allowing fine control, including 6 actions: move forward/backward, turn left/right, and turn left/right + move forward. The environment run at 60 frames-per-second, and the extrinsic reward is achieved by reaching apple (worth + 1 point) and goal (worth + 10 points) in the environment. If the goal is reached, the agent is respawned to a new start location, and the episode does not end until a fixed amount of time expires.

#### 4.1.2. Baselines

We compared our method to a set of baselines that rely on intrinsic motivation to guide exploration. The simplest baseline was the basic RL algorithm Trust Region Policy Optimization (TRPO) [35], which uses heuristic *ε* − greedy strategy to encourage exploration. Then, we take VIME [15] as a comparison object; this method perceives dynamic changes of environment based on Bayesian Neural Network (BNN) and obtains exploration policy through maximizing such information gain. The third baseline is a classifier-centered approach EX2 [16], and its novelty detection of exploration relies entirely on a discriminatively trained exemplar model. Finally, as a sanity check, we reproduce the state-of-the-art curiosity method ICM [17] in our experiment.

#### 4.1.3. Model Implementation

The details of the architecture of our exploration model are as follows. It has two layers of CNN: the first one with 8 × 8 filters applied with stride 4 × 4 and 16 feature maps and the second with 4 × 4 filters with stride2 × 2 and 32 feature maps. Next there is a fully connected layer with 256 units, and all three layers are followed by a ReLU nonlinearity unit. After that, an LSTM layer with 256 units uses the CNN's encoded observation, previous action, and previous reward as input, and the policy and value function are linear projections of the LSTM layer output.

For the TC-network, the inputs are two observations, each processed by a ResNet-18 encoder and producing 512-dimensional feature vector. The TC-network concatenates these features firstly and then puts them to a fully connected network with four hidden layers, each equipped with 512 units and a ReLU nonlinearity unit, to predict if the two observations are adjacent or not.

#### 4.1.4. Hyperparameters

In the exploration process, we chose the commonly used A3C algorithm as the basic RL approach and used 84 × 84 RGB observation that samples at intervals of three frames (every action is repeated 4 times) as input. Eight workers were equipped with noncentered RMSProp to interact with the environment setting in parallel. The learning rates were sampled from a log-uniform distribution between 0.0001 and 0.005, and the entropy costs were sampled from a log-uniform distribution between 0.0005 and 0.01.

The inputs of TC-network are two RGB images at the resolution of 160 × 120 pixels, and all the training data are generated by the agent itself. We randomly sample a minibatch of 64 observation pairs from the replay buffer *B* during training and perform an update using the Adam optimizer [36] with a learning rate *λ*=0.0001.

### 4.2. Parameter Selection Experiment

We are interested in an agent that can explore the environment spontaneously. However, before testing the performance of our approach, some parameters need to be set up in advance. These parameters mainly involve two aspects: one is the training details in TC-network; the other one is the key element about intrinsic motivation; we will confirm them in the maze shown in Figure 8.

#### 4.2.1. Sample Separation Parameter

In the process of training TC-network, a threshold *k* is required to separate positive from negative sample pairs. To obtain suitable training samples, we conduct an experiment that make *k* vary from 1 to 10 and show its influence to TC-networks and memory buffer. The training results (1.5 M interaction quantity) of TC-network are averaged over the top 5 random hyperparameters, and the proportion of observations stored in memory buffer (POSM) are calculated based on the corresponding TC-network and 30 random observation sequences.  Table 1 shows that the training effect of TC-network is closely related to the difference between positive and negative samples. In the beginning, due to the small difference between samples, the accuracy of TC-network is low. Then, the prediction ability goes up with the increase of *k*, but when the threshold is greater than a value, the accuracy falls again. As we expected, the number of stored observations drops off with the increase of *k* and augments again when the prediction ability of TC-network reaches a bottleneck.

The experiment results put us in a dilemma because TC-network is the key to generate intrinsic motivation; we must keep it in good condition. However, we also support storing as few observations as possible during the interaction. After careful consideration, we choose the data separated by 4-time steps as training samples.

#### 4.2.2. Interaction Quantity Parameter

Except for threshold *k*, the interaction quantity with the environment is another important parameter in the pretraining phase. In our method, the sample complexity includes two parts: pretraining and online learning. The exploration behavior is finished by online learning and with no need for care about the sample size, but such situation is opposite in the pretraining part. The relationship between the amount of interaction and network performance is shown in Table 2, and the results are averaged over the top 5 random hyperparameters. As Table 2 demonstrates, the accuracy of TC-network goes up with the expansion of training data while decreasing when the network is overfitting. In order to have efficient training and maintain good performance of the network, the interaction quantity of pretraining is set as 2.5 M.

In conclusion, the TC-network can learn useful controllers based on trajectories of a randomly acting agent and use it to create intrinsic motivation. However, since all the samples in pretraining stage come from the same environment, it inevitably leads to a lack of generality in TC-network. So, in the subsequent exploration process, we will collect data from different environments and conduct second training for TC-network.

#### 4.2.3. Intrinsic Motivation Parameter

Our intrinsic motivation *r*_*t*_^*i*^ is an augmented reward; it consists of two types of novelty bonus. In order to tradeoff the influence between the bonus, we test the effect of different parameter groups, which setup *α*+*β* ≡ 1 and sample them in the same interval (0.1), and mainly demonstrate two results: the episode reward (novelty bonus generated by the agent within 1800 time steps) and the amount of interaction required to encode the environment. The results are averaged over the top 5 random hyperparameters and are summarized in Figure 9 after data normalization (take the lowest result as standard). As Figure 9 demonstrates, relying on one type of novelty bonus, where *α*, *β*=(0.0, 1.0) or *α*, *β*=(1.0, 0.0), the agent is able to generate various exploration behavior. However, their exploration efficiency is lower than the agents that simultaneously use the two types of novelty bonuses, which is why these agents need more interaction to encode the environment. Meanwhile, we can interpret the experiment results from the composition of intrinsic motivation. Our intrinsic motivation includes two parts and each of them focuses on a direction: the count-based method pays attention to the novelty bonus of the environment that has been explored, encouraging the agent to reach the rarely visited states; the temporal distance method concentrates on calculating the novelty bonus of unexplored area and trying to push the agent to a distant place. Therefore, it is beneficial to use them together to guide exploration.

Among all the agents, the one equipped with the parameter group *α*, *β*=(0.2, 0.8) shows the best exploration efficiency and requires fewer interaction to encode the environment, so we select *α*=0.2 and *β*=0.8 in the following experiment. In addition, unlike the pretraining stage, the agent no longer acts randomly but learns an exploration policy in the environment (Figure 8); this is the basis to conduct fine-tuning method in other mazes.

### 4.3. Exploration Experiment

The goal of the experiment was to quantitatively evaluate the exploration performance of different approaches and learning patterns. The test environment is shown in Figure 10. The structure of Maze-1 and Maze-2 was inspired by spatial cognition experiments in rodents, the former consisting of three paths of different lengths, and the latter have a central corridor and six arms. Maze-3 is a common maze that includes various obstacles. There was no extrinsic reward (such as goal or fruit) available in these mazes.

The performance of each method was evaluated by a uniform count-based reward, which was calculated based on the area explored by the agent within an episode. The learning process was presented as an episode reward/training step diagram (results are averaged over the top five random hyperparameters), within the time limit of 7200 steps (equivalent to two minutes), and the agent had to explore the environment as much as possible. Every time the episode is done, the agent was respawned into a new location and had to explore the environment again.

#### 4.3.1. Learning Exploration from Scratch

In our first set of experiments, the entire exploration policy was learned from scratch. In addition, because the TC-network needs an extra 2.5 M of data to finish pretraining, for a fair comparison, we shift the curves for our method by the number of environment steps to train it.

By analyzing the training curves, shown in Figure 11, we can draw several conclusions. First, the VIME method, which achieves good results on simple, clean images in the Atari games, struggles in all test mazes. This is because the BNN is insufficient to support a dynamic model that is built from a first-person view, in which the agent shows reactive behavior in the learning process. The worst case occurs in Maze-1, where the area explored by VIME is even smaller than the randomly acting agent. Second, compared with VIME, the EX2 is more applicable in challenging image-based environments. It generates coherent exploration behavior and guides the agent to reach alcoves of the end in Maze-2. However, EX2 requires a good deal of interaction to train the exemplar model, resulting in the reward it obtained being lower than 300 in the early training stage. Owing to the limited ability of the classifier, as the structure of mazes becomes more complex, more areas lose their deserved novelty bonus and are neglected by the agent. Finally, the exploration policy achieved by ICM and our method greatly exceeds that of prior exploration techniques, thereby proving that these methods are suitable to high-dimensional continuous state spaces. The difference in performance between them is more obvious in Maze-3. Because there are many obstacles and hidden areas within Maze-3, relying on prediction error to guide exploration can easily produce a dead zone. Meanwhile, our method, which generates intrinsic motivation based on episode memory, can push the agent to explore every corner in the environment. One last thing to note is that, despite ICM and our method get almost equal rewards in Maze-1 and Maze-2, our method is able to push the agent to reach distant state and discover more areas with the same interaction.

Table 3 lists exploration indicators, including the achieved reward, the maximum exploration ratio (MER) within an episode, and the interaction quantity required to encode the environment (IQRE). The IQRE metric demonstrates the exploration efficiency of different approaches, which are calculated using preobtained environmental features and observations stored during the exploration of the agent. As shown in Table 3, both the reward and explored area increase with the improvement of exploration efficiency. To our surprise, the basic exploration method TRPO, whose behavior depends primarily on random actions, still covers half of Maze-1 and obtains the reward almost equal to VIME in Maze-2. For the second baseline, the agent walks like an aimless human (such as wall-following behavior) and is unable to explore the environment consciously, because the VIME method lacks appropriate inference about environment dynamics. The following methods show better performance in high-dimensional visual spaces. EX2 achieves at least 70% coverage compared to the first two mazes and makes the agent reach more than 50% area in Maze-3. The ICM model guides the agent to obtain complete memory of Maze-1 and Maze-2, but it needs substantial interaction to stabilize exploration behavior, and such policy is not guaranteed in Maze-3. Compared with previous methods, our approach maintains an effective exploration policy across different mazes and uses it to push the agent to cover the environment. In terms of exploration efficiency and the amount of training data required for policy convergence, our method is superior to others, and such phenomena are evident in Maze-1 and Maze-2.

In addition, it shown in Table 4 that the accuracy of the pretrained TC-network declines rapidly in a new environment. If we make no adjustments to it, the performance of subsequent exploration will be affected. We also find that training the TC-network for each maze is not a wise choice, because such a targeted method will significantly increase the cost of pretraining and put off the process of creating intrinsic motivation, although it achieves better prediction ability. Therefore, we fine-tune the secondary training for the TC-network. This online method can randomly sample training data from each test maze in the process of learning control policy. In fact, the generalization training reduces the accuracy of TC-network, but such reduction is acceptable. Meanwhile, the training process can be completed within 2.5 M interaction (equal to the pretraining stage) and does not prevent the agent from exploring the mazes.

#### 4.3.2. Learning Exploration with the Fine-Tuning Method

In the previous section, we showed how the ICM model and our approach can efficiently guide the agent in exploring the environment. However, such an exploration policy is learned from scratch. We want to know whether these methods could be trained with fine-tuning. To answer this question, we used the exploration policy that was obtained in Section 4.2.3 (trained in the environment shown in Figure 8) as initial input and then used the fine-tuning method to train ICM and our approach in each maze. At the same time, we studied the effect of extrinsic reward on learning exploration policy.

Figure 12 shows how using the fine-tuning method to train the agent can end the random behavior sooner and achieve an effective exploration policy in new environments, but the training effect varies in different mazes. As shown in Table 5, there is no marked difference between learning from scratch or fine-tuning in Maze-1, either from the achieved reward or the amount of interaction required to cover the environment. However, their learning curves show that because the structure of Maze-1 is relatively simple, learning from scratch is an efficient way to achieve exploration policy. They also show that the fine-tuning method, whose initial parameters include behaviors such as wall-walking, obstacle avoidance, and turning a corner, makes some mismatches in the early training stage. In Maze-2, compared with learning from scratch, the fine-tuning method significantly speeds up the training efficiency of ICM and enables it to use less interaction to converge the policy, but such improvement is not witnessed in our method. The role of fine-tuning can be better illustrated in Maze-3, and the effects manifest themselves in two aspects: that the exploration performance of ICM has improved again and that the amount of interaction needed to encode the environment has been further reduced. Overall, the improvement brought about by fine-tuning is more helpful for ICM, while our method shows stability and scalability across different learning patterns.

Next, we put extrinsic rewards in each maze and retrained ICM and our method with fine-tuning. The extrinsic reward is in the form of goal (worth + 10) and apple (worth + 1), and their location is fixed in an episode and varies randomly between episodes. If the goal is reached, the agent is respawned to a new start location and has to explore the maze again, and the performance of each method is measured by the uniform count-based reward. The experiment results are shown in Figure 13 and Table 6. It can be seen that, compared to the former method, using extrinsic reward to conduct the fine-tuning results in more negative effects, it not only slows down the training process, but also confuses exploration and navigation. Such damage to performance is rooted in the driving force, which results in the states, including extrinsic reward, becoming attractive during exploration and the agent wanting to reach it consistently. In addition, because the agent will be reset to a new location when it reaches the goal, the purpose of fine-tuning seems to be finding the goal instead of exploring the environment. This is why the agent can quickly get a good reward in the early training period but still need more interaction to complete the exploration. This phenomenon is particularly obvious in Maze-1 and Maze-2, while the worst case occurs in Maze-3, because there is no one method trained by fine-tuning that can guide the agent to cover the environment within an episode.

#### 4.3.3. “Noisy-TV” Experiment

In the previous section, we observed that the ICM method is superior to other baselines and achieves nearly the same performance as our method in the first two test mazes. However, the “couch-potato” issue, which appears in the “noisy-TV” experiment, is still a challenge of such a prediction-based curiosity method. While our method relies on the agent's observation and memory to guide exploration, the goal of this experiment is to provide additional evidence to verify whether it is more robust to stochastic objects.

The “noisy-TV” experiment is implemented as follows. In all test environments, the TV is on the head-on display of the agent, and its location is fixed within an episode. An image at resolution of 21 × 21 is shown on the TV screen at every time step, independently from the agent's actions, and each pixel in the image is sampled uniformly from [0,255].

The experiment results that appear in Figure 14 and Table 7 show that the performance of ICM and our method both deteriorated after adding the source of stochasticity, but that ICM was more severely affected. The ICM exhausted its curiosity very quickly and exploration was stalled when learning from scratch, while the fine-tuning method was able to promote exploration to some extent, but the obtained policy was not satisfactory. It can be seen that some parts of state space simply cannot be modeled, like the “noisy-TV” in this experiment. Their prediction error will remain high and show an irresistible attraction to the ICM model, thereby making the agent fall into a curiosity trap and deteriorate into undesired behavior. Obviously, the images of “noisy-TV” are inconsequential to exploration, and the agent's continued curiosity about them is useless. In our approach, the agent seeks out the curiosity based on memory instead of prediction. Relying on a comparison to the past, the agent will not maintain curiosity about such stochastic objects and will overcome the “couch-potato” issues. The experiment results show that our method can explore the environment reasonably well and obtain the complete memory of all test mazes, although the presence of “noisy-TV” slows down the learning speed.

## 5. Conclusion

In this work, we proposed an autonomous exploration method based on deep reinforcement learning and the concept of intrinsic motivation. One component of our method has the objective of creating intrinsic motivation while the other has the objective of learning exploration policy, and they are designed to work together. Our experiment results and analysis highlight the role of intrinsic motivation and training method in learning exploration policy. We also examine the agent's performance in an environment that includes stochastic objects.

Our approach is inspired by the behavior of curiosity in animals, which enables them to explore the environment without any extrinsic reward. For AI agents, to accomplish the autonomous exploration with raw visual inputs, we use deep reinforcement learning as the basic framework and allow the agent to create rewards for itself. Considering the limitations of prediction-based exploration methods, our intrinsic motivation is calculated based on episode memory and include two types of novelty bonuses. This enables our approach to outperform the existing methods in 3D maze-like environments and gives it better ability to handing stochastic objects.

Although our approach successfully learns exploration policy from visual inputs, its performance would be limited in very large environments, owing to the capacity of the single-layer LSTM and the memory buffer. In the future, it is necessary to increase the capacity of our exploration model by adding LSTMs or using external memories. Furthermore, we believe it would be intriguing for future work to migrate our method to the real world and compare it with vision-based simultaneous localization and mapping (SLAM) approaches.

## Figures and Tables

**Figure 1:** AC algorithm flow chart.

**Figure 2:** The A3C algorithm flow chart.

**Figure 3:** Nav A3C model.

**Figure 4:** TC-network model.

**Figure 5:** Calculation process of intrinsic motivation.

**Figure 6:** Exploration model.

**Figure 7:** Simulation environment. (a) Go forward. (b) Apple. (c) Goal. (d) Door.

**Figure 8:** Parameter selection environment.

**Figure 9:** Experiment results of the reward function parameter.

**Figure 10:** Top-down view of test mazes. (a) Maze-1. (b) Maze-2. (c) Maze-3.

**Figure 11:** Experiment results of learning exploration from scratch. (a) Learning curves in Maze-1. (b) Learning curves in Maze-2. (c) Learning curves in Maze-3.

**Figure 12:** Experiment results of learning exploration with fine-tuning method (no extrinsic reward). (a) Learning curves in Maze-1. (b) Learning curves in Maze-2. (c) Learning curves in Maze-3.

**Figure 13:** Experiment results of learning exploration with fine-tuning method (exist extrinsic reward). (a) Learning curves in Maze-1. (b) Learning curves in Maze-2. (c) Learning curves in Maze-3.

**Figure 14:** Experiment results of “noisy-TV.” (a) Learning curves in Maze-1. (b) Learning curves in Maze-2. (c) Learning curves in Maze-3.

**Table 1:** Experiment results of sample separation parameter.

*k*	TC-network (%)	POSM (%)
1	88.68	31.25
2	91.53	22.34
3	93.06	16.27
4	92.32	12.51
5	90.87	11.63
7	86.59	12.48
10	81.93	12.65

**Table 2:** Experiment results of interaction quantity parameter.

Sample size	TC-network (%)
300 K	80.35
500 K	82.42
1 M	87.95
2.5 M	92.63
5 M	91.02

**Table 3:** Experiment results of learning exploration from scratch.

Environment	Method	Reward	MER (%)	IQRE
Maze-1	TRPO	327.36	55.29	N/A
	VIME	321.14	53.58	N/A
	EX2	489.27	82.43	N/A
	ICM	584.59	100.00	7.93
	Ours	586.32	100.00	4.72
Maze-2	TRPO	232.47	41.02	N/A
	VIME	228.34	39.98	N/A
	EX2	425.73	74.56	N/A
	ICM	567.28	100.00	8.07
	Ours	571.87	100.00	5.15
Maze-3	TRPO	243.49	41.73	N/A
	VIME	276.54	47.82	N/A
	EX2	339.62	58.35	N/A
	ICM	532.27	91.64	N/A
	Ours	579.65	100.00	6.54

**Table 4:** The secondary training results for TC-network.

Method	Environment	TC-network (%)
Pretraining	Parameter selection	92.36
	Maze-1	84.52
	Maze-2	85.14
	Maze-3	78.32
Targeted training	Maze-1	93.16
	Maze-2	92.67
	Maze-3	92.03
Generalization training	Maze-1/Maze-2	90.89
	Maze-1/Maze-3	91.35
	Maze-2/Maze-3	90.62
	Maze-1/Maze-2/Maze-3	90.28

**Table 5:** Experiment results of learning exploration with fine-tuning method (no extrinsic reward).

Environment	Method	Reward	MER (%)	IQRE
Maze-1	ICM + scratch	584.59	100.00	7.93
	Ours + scratch	586.32	100.00	4.72
	ICM + fine-tuning	585.16	100.00	7.58
	Ours + fine-tuning	585.45	100.00	5.14
Maze-2	ICM + scratch	567.28	100.00	8.07
	Ours + scratch	571.87	100.00	5.15
	ICM + fine-tuning	566.34	100.00	6.49
	Ours + fine-tuning	568.25	100.00	4.81
Maze-3	ICM + scratch	532.27	91.64	N/A
	Ours + scratch	579.65	100.00	6.54
	ICM + fine-tuning	573.49	100.00	7.23
	Ours + fine-tuning	572.86	100.00	4.73

**Table 6:** Experiment results of learning exploration with fine-tuning method (exist extrinsic reward).

Environment	Method	Reward	MER (%)	IQRE
Maze-1	ICM + scratch	584.59	100.00	7.93
	Ours + scratch	586.32	100.00	4.72
	ICM + fine-tuning	583.74	100.00	9.13
	Ours + fine-tuning	586.56	100.00	7.24
Maze-2	ICM + scratch	567.28	100.00	8.07
	Ours + scratch	571.87	100.00	5.15
	ICM + fine-tuning	514.63	89.46	N/A
	Ours + fine-tuning	569.44	100.00	6.83
Maze-3	ICM + scratch	532.27	91.64	N/A
	Ours + scratch	579.65	100.00	6.54
	ICM + fine-tuning	483.16	82.95	N/A
	Ours + fine-tuning	542.68	92.63	N/A

**Table 7:** Experiment results of “noisy-TV.”

Environment	Method	Reward	MER (%)	IQRE
Maze-1	ICM + scratch	315.62	53.86	N/A
	Ours + scratch	582.74	100	7.58
	ICM + fine-tuning	374.52	64.05	N/A
	Ours + fine-tuning	586.43	100	8.67
Maze-2	ICM + scratch	279.68	48.71	N/A
	Ours + scratch	565.32	100	6.93
	ICM + fine-tuning	317.54	56.18	N/A
	Ours + fine-tuning	566.73	100	7.75
Maze-3	ICM + scratch	362.49	63.28	N/A
	Ours + scratch	577.86	100	7.69
	ICM + fine-tuning	305.47	54.72	N/A
	Ours + fine-tuning	572.63	100	8.12

## Data Availability

We did not use any specific dataset, and all the experiment data were from the public data platform, DMLab.
